# Biomechanical Investigation of the Posterior Pedicle Screw Fixation System at Level L4-L5 Lumbar Segment with Traditional and Cortical Trajectories: A Finite Element Study

**DOI:** 10.1155/2022/4826507

**Published:** 2022-03-28

**Authors:** Alafate Kahaer, Zhihao Zhou, Julaiti Maitirouzi, Shuiquan Wang, Wenjie Shi, Nueraihemaiti Abuduwaili, Xieraili Maimaiti, Dongshan Liu, Weibin Sheng, Paerhati Rexiti

**Affiliations:** ^1^Department of Spine Surgery, The First Affiliated Hospital of Xinjiang Medical University, Urumqi 830054, Xinjiang, China; ^2^College of Mechanical Engineering, Xinjiang University, Urumqi 830054, Xinjiang, China; ^3^Department of Anatomy, College of Basic Medicine, Xinjiang Medical University, Urumqi 830054, Xinjiang, China; ^4^Xinjiang Medical University, Urumqi 830054, Xinjiang, China; ^5^Department of Imaging Center, The First Affiliated Hospital of Xinjiang Medical University, Urumqi 830054, Xinjiang, China

## Abstract

There is no detailed biomechanical research about the hybrid CBT-TT (CBT screws at cranial level and TT screws at caudal level) and TT-CBT (TT screws at cranial level and CBT screws at caudal level) techniques with finite element (FE) method. Therefore, the purpose of this study was to evaluate and provide specific biomechanical data of the hybrid lumbar posterior fixation system and compare with traditional pedicle screw and cortical screw trajectories without fusion, in FE method. Specimens were from the anatomy laboratory of Xinjiang Medical University. Four FE models of the L4-L5 lumbar spine segment were generated. For each of these, four implanted models with the following instruments were created: bilateral traditional trajectory screw fixation (TT-TT), bilateral cortical bone trajectory screw fixation (CBT-CBT), hybrid CBT-TT fixation, and hybrid TT-CBT fixation. A 400 N compressive load with 7.5 Nm moments was applied so as to simulate flexion, extension, left lateral bending, right lateral bending, left rotation, and right rotation, respectively. The range of motion (ROM) of the L4-L5 segment and the posterior fixation, the von Mises stress of the intervertebral disc, and the posterior fixation in four implanted models were compared. CBT-TT displayed a lower ROM of the fixation segment (3.82 ± 0.633°) compared to TT-TT (4.78 ± 0.306°) and CBT-CBT (4.23 ± 0.396°). In addition, CBT-TT showed a lower ROM of the posterior fixation (0.595 ± 0.108°) compared to TT-TT (0.795 ± 0.103°) and CBT-CBT (0.758 ± 0.052°). The intervertebral disc stress of CBT-TT (4.435 ± 0.604 MPa) was lower than TT-TT (7.592 ± 0.387 MPa) and CBT-CBT (6.605 ± 0.600 MPa). CBT-TT (20.228 ± 3.044 MPa) and TT-CBT (12.548 ± 2.914 MPa) displayed a lower peak von Mises stress of the posterior fixation compared to TT-TT (25.480 ± 3.737 MPa). The hybrid CBT-TT and TT-CBT techniques offered superior fixation strength compared to the CBT-CBT and TT-TT techniques.

## 1. Introduction

The pedicle screw fixation technique has become the mainstay for the treatment of various lumbar diseases, providing considerable biomechanical stability [1, 2]. However, it is common for complications to occur, including screw loosening and breaking, which cause posterior fixation failure due to insufficient purchase of the pedicle screw-bone interface resulting from reduced bone mineral density and sparse bone. This condition is more common in elderly patients with osteoporosis [3, 4]. Some studies suggested that postoperative spinal stability could be maintained by improving the purchase of posterior fixation in elderly patients with osteoporosis [4].

To increase the purchase and stability of the screw-bone interface and obtain superior posterior fixation strength in patients with osteoporosis or lumbar revision surgery, numerous attempts have been made by researchers over the years, from the shape design of screws to the curing of screw tracks, including screw augmentation with allograft or cement [5, 6], expandable pedicle screws [7, 8], and screw surface hydroxyapatite coating [9, 10]. However, these have some limitations in the clinic because of the disadvantages of potential safety hazards, high price, and complications [11, 12].

Santoni et al. [13] proposed the cortical bone trajectory (CBT) in 2009, with a mediolaterally and a caudocranially directed path through the pedicle. CBT displayed a 30% increase in uniaxial yield pullout load [13] and a 1.7 times higher torque [14] compared with that for the traditional trajectory (TT) in the cadaveric lumbar spine. Additionally, screw insertion through a medial starting point avoids wide exposure of the superior facet joint and minimizes muscle dissection, providing minimal invasiveness and reducing the incidence of adjacent segment disease (ASD) [15]. However, CBT screws also have many limitations [16, 17]. Particularly in traditional transforaminal lumbar interbody fusion (TLIF), the lateral recess of the lower lumbar spine frequently requires decompression, which has a certain impact on CBT screw placement. In single-segment fixation, pars fracture is contraindicated when using cortical bone trajectory screw, which needs pedicle screw for alternative fixation, whereas hybrid techniques could avoid this problematic situation. Human cadaveric study and clinical trials have reported on the hybrid CBT-TT technique [18–20], but limited in stiffness and pullout strength [20], no detailed biomechanical research has been published considering the biomechanical properties of the hybrid CBT-TT and TT-CBT techniques. In this paper, we further evaluate the biomechanical properties, the range of motion (ROM) of the fixation segment and the posterior fixation, the von Mises stress of the intervertebral disc, and the posterior fixation, of hybrid techniques in six different working conditions by finite element (FE) analysis in combination with the practical application of the hybrid techniques to provide a mechanical theoretical reference for the clinic.

## 2. Materials and Methods

### 2.1. Model Development of the L4-L5 Lumber Spine

High-resolution computed tomography (CT) data (AQUIRRON 16, PHILIPS, Netherlands) of the L4 to L5 vertebrae in four lumbar specimens (two males and two females) from the Anatomy Teaching-Research Office of Xinjiang Medical University were acquired. The mean age of the four specimens was 71, ranging from 64 to 77 years, and they were free from lumbar fracture, tumor, tuberculosis, and malformation. Among them, the L5 vertebra of one specimen had an isthmus breakage and spondylolisthesis. Anatomical three-dimensional (3D) models of the L4–L5 lumbar spine vertebrae were generated using mimics 16.0 (Materialize, Leuven, Belgium). The models were embedded into hypermesh 18.0 (3D Systems Corporation, Rock Hill, South Carolina, USA) for further operation, including repairing the damaged and missing areas, retriangulation and smoothing of the polygon mesh, making triangles more uniform in size, and generating a nonuniform rational B-spline (NURBS) surface on the object. This meshing process was performed for screws implanted into lumbar spine together with the lumbar spine model itself to ensure the continuity of the mesh. Cortical bone was defined as a 0.5 mm thickness outward from the outer layer of the cancellous bone [21]. The areas of the screw insertions were the focus of this study; thus, appropriate mesh refinement was performed for these sites to ensure the precision of the results. Meshed models were finally generated with a maximum size of 1.5 mm and a minimum size of 0.5 mm. Eventually, the meshed models were processed using ABAQUS 2019 (ABAQUS, Providence, Rhode Island, USA) to set the material properties of the vertebral body, intervertebral disc, and posterior fixation. Although the various parts of the bone model were strictly nonlinear, superelastic materials, they were simplified as linear elastic and homogeneous materials for FE analysis in this study. Therefore, we also defined the material properties of each component in the category of elastic materials (Table 1). The relationship between the L4 and L5 vertebral bodies and the intervertebral disc was defined as the mutual contact, and a more rigid intervertebral disc was selected as the active surface, using a face-to-face correspondence, with a friction coefficient of 0.08, and a contact mode without separation was adopted. The contacts between the reference point and the vertebra were defined using “contact” constraint. Finally, the parts were assembled into a complete L4-L5 model.

### 2.2. Construction of Surgical Models

Four different posterior fixations used in this study were as follows: (1) TT-TT, TT screws at the cranial and caudal levels (Figure 1(a)); (2) CBT-CBT, CBT screws at the cranial and caudal levels (Figure 1(b)); (3) CBT-TT, CBT screws at the cranial level and TT screws at the caudal level (Figure 1(c)); (4) TT-CBT, TT screws at the cranial level and CBT screws at the caudal level (Figure 1(d)). A total of 16 finite element models were generated based on data from four anatomical specimens. Accuracy of the placement of screws with the same trajectory was strictly controlled in all models. The starting point for CBT was located at the lateral aspect of the pars interarticularis projecting in the 5 o'clock orientation in the left pedicle and the 7 o'clock orientation in the right pedicle, using the clock face for orientation [22]. CBT screws were inserted 10° laterally in the axial plane and 25° cranially in the sagittal plane [23] (Figure 1(f)). Titanium-based rods measured 5.5 mm in diameter; the TT screws had a length of 45 mm and a diameter of 6.0 mm; the CBT screws had a length of 35 mm and a diameter of 4.5 mm. The lower edge of the L5 vertebral body was fully fixed to constrain the motion in six directions throughout the analysis to ensure that there was no displacement or rotation with the force applied on the L4 vertebral body. To apply compressive load and torque, a reference point was created in the center of the superior surface of the L4 vertebral body.

### 2.3. Biomechanical Analysis

The axial displacement of the model was calculated by applying compressive loads of 500, 1000, 1500, and 2000 N to the reference points on the superior surface of the L4 vertebra, respectively, and compared with the in vitro experimental results of Markolf [24], Virgin [25], and Brown et al. [26] to verify the reliability and accuracy of the model in the present study.

To achieve a clinical simulation, a compressive load of 400 N and a torque of 7.5 Nm were applied to the reference point on the superior surface of the L4 vertebra to simulate flexion, extension, left lateral bending, right lateral bending, left rotation, and right rotation, respectively. The ROM of the L4-L5 segment and posterior fixation, von Mises stress of the intervertebral disc, and posterior fixation were recorded to make a biomechanical comparison of the hybrid CBT-TT and TT-CBT techniques with the TT-TT and CBT-CBT techniques. In the present study, the von Mises stress was selected as the equivalent stress for the disc and posterior fixation.

### 2.4. Statistical Methods

SPSS 22.0 software was used for data analysis and processing. The data distribution was expressed as the mean ± standard deviation. The difference analysis was performed by one-way analysis of variance (ANOVA). When there were statistical differences in different indicators, the Bonferroni pairwise comparison method was used as the post hoc test. *P* < 0.05 was considered statistically significant for all analyses.

## 3. Results

### 3.1. Validation of the Intact Model

The final model contained 195,858 nodes and 58,085 elements, and the axial displacements of the models under the four increasing compressive loads were 0.336, 0.654, 0.813, and 1.132 mm, respectively (Figure 2). The results of this study were in good agreement with previous in vitro tests [24–26]. Therefore, the four intact models were included for further biomechanical analysis. The comparison between the results of the current study and the previous studies showed that the ROMs of the L4-L5 segments were within the range of those previous studies [27–30] (Figure 3).

### 3.2. Range of Motion of the L4-L5 Segment

The ROMs of the intervertebral disc of CBT-TT and TT-CBT were significantly reduced in comparison with TT-TT (*P* ≤ 0.013), except for left rotation (*P* ≥ 0.113), and with no differences in each of the six conditions (*P* ≥ 0.106) in comparison to CBT-CBT. Among the four fixation models, the highest ROM at the L4–L5 level was found for TT-TT, followed by CBT-CBT, TT-CBT, and CBT-TT (Figure 4). In comparison with the ROMs in TT-TT, those in CBT-TT were decreased by 16% in flexion, 18% in extension, 27% in left lateral bending, 37% in right lateral bending, 18% in left rotation, and 20% in right rotation. In addition, the ROMs in TT-CBT were decreased by 18% in flexion, 19% in extension, 25% in left lateral bending, 41% in right lateral bending, 17% in left rotation, and 19% right rotation, compared with TT-TT.

### 3.3. Range of Motion of Posterior Fixations

The ROMs of posterior fixation of CBT-TT and TT-CBT were significantly reduced in comparison to TT-TT (*P* ≤ 0.001), except for the left and right rotations (*P* ≥ 0.115, *P* ≥ 0.342, respectively). In flexion, extension, and right lateral bending, the ROMs of posterior fixation were significantly decreased in comparison to CBT-CBT (*P* ≤ 0.021). Among the four fixation models, the highest ROM was found for TT-TT, followed by CBT-CBT, CBT-TT, and TT-CBT (Figure 5). In comparison with TT-TT, the ROMs in TT-CBT were decreased by 36% in flexion, 40% in extension, 15% in left lateral bending, 26% in right lateral bending, 31% in left rotation, and 11% in right rotation. In addition, ROMs in CBT-TT were decreased by 38% in flexion, 40% in extension, 14% in left lateral bending, 24% in right lateral bending, 35% in left rotation, and 25% in right rotation, compared with TT-TT.

### 3.4. The Stress of the Intervertebral Disc

The stress distributing contours of the discs in the fixation segment could provide a visual comparison of the stabilizing ability among the four fixations (Figure 6). CBT-TT displayed the least stressing contours in the left and right rotations compared to the counterparts. TT-CBT provided the highest load-sharing ability to the fixed segment, followed by CBT-TT, CBT-CBT, and TT-TT, particularly in left rotation. In all conditions, the disc stresses of CBT-TT and TT-CBT were significantly decreased compared with the counterparts (*P* ≤ 0.021), while the disc stress of TT-CBT was significantly decreased in comparison with CBT-TT in flexion and extension (*P* ≤ 0.008). The highest ROM was found for TT-TT, followed by CBT-CBT, TT-CBT, and CBT-TT (Figure 7). In comparison with TT-TT, the ROMs in TT-CBT were decreased by 53% in flexion, 47% in extension, 31% in left lateral bending, 31% in right lateral bending, 41% in left rotation, and 41% in right rotation. In addition, ROMs in CBT-TT were decreased by 43% in flexion, 42% in extension, 35% in left lateral bending, 36% in right lateral bending, 40% in left rotation, and 40% in right rotation, compared with TT-TT.

### 3.5. The Stress of the Posterior Fixations

A similar change in the maximal von Mises stress in the posterior fixations was observed, with the highest stress of the fixations found in TT-TT, followed by CBT-CBT, CBT-TT, and TT-CBT (Figure 8). As can be seen in Figure 9, the maximal von Mises stress on the screw hub and the rod of CBT-TT and TT-CBT were reduced in all working conditions. In comparison with TT-TT, the von Mises stress of posterior fixation in TT-CBT significantly decreased (*P* ≤ 0.05), except for left lateral bending, and this in CBT-TT was also significantly decreased (*P* ≤ 0.048), except for lateral bending and right rotation. A typical minimal von Mises stress of TT-CBT is presented in Figure 9. Compared with TT-TT, the mean value of the von Mises stress in TT-CBT was decreased by 35% in flexion, 23% in extension, 36% in left lateral bending, 51% in right lateral bending, 30% in left rotation, and 29% in right rotation, which was decreased by 34% in flexion, 28% in extension, 23% in left lateral bending, 20% in right lateral bending, 18% in left rotation, and 9% in right rotation in CBT-TT, compared with TT-TT. The maximum values of the von Mises stress in TT-CBT fixation were 65.4 MPa in flexion, 68.4 MPa in extension, 24.5 MPa in left lateral bending, 16.7 MPa in right lateral bending, 29.6 MPa in left rotation, and 28.64 MPa in right rotation, respectively.

## 4. Discussion

FE analysis has been increasingly applied in spinal-related biomechanical studies [23, 31, 32] and is suitable for single-stage and multistage models to investigate the biomechanical properties of posterior fixation techniques. It has the advantages of flexibly moderating the relevant parameters under the same conditions for multiple and fair comparisons and analyses. Additionally, it can reduce the bias rate. From a biomechanical point of view, the forces of transverse processes, vertebral plates, and facet joints converge at the pedicle, that is, as the “force nucleus” of the vertebral body [33]. CBT screws achieve better fixation strength by maximizing the contact area of the screw threads with cortical bone in the “force nucleus,” including the dorsal cortical bone at the insertion, the medially oriented posterior pedicle wall, the laterally oriented anterior pedicle wall, and the curvature of the vertebral body wall [14]. However, it was not the best fixation technique. Takata et al. [18] first proposed a hybrid CBT-TT technique and applied it to patients with degenerative spondylolisthesis, which could reduce the peeling of soft tissue and the incision length. Chiu et al. [19] demonstrated that the mean Numeric Rating Scale and Oswestry Disability Index scores were significantly improved, the damaged anterior column could be debrided and reconstructed, and spinal stabilization could be achieved when applying the hybrid CBT-TT technique in patients with spondylodiskitis. In addition to CBT-TT, we proposed the hybrid TT-CBT technique for patients with lumbar spondylolisthesis. There have been previous mechanical studies related to CBT screws that have focused on noninferior toggle and pullout strength in direct comparison to TT screws [13, 14, 32]. However, no research has been published that addresses segmental stability when comparing the hybrid CBT-TT and TT-CBT with TT-TT and CBT-CBT techniques.

In the present study, a single-stage lumbar FE model was selected to investigate the biomechanical stability of osteoporotic lumbar spine models in different posterior fixation techniques. Several previous biomechanical studies by Matsukawa et al. [23, 34] demonstrated that CBT-CBT has a significantly superior vertebral stability in flexion-extension and inferior stability in lateral bending compared to TT-TT. Meanwhile, the present study showed that there was a lower ROM of L4–L5 segment in CBT-CBT compared to TT-TT in flexion (CBT-CBT: 5.44 ± 0.153°, TT-TT: 6.73 ± 0.477°) and extension (CBT-CBT: 5.80 ± 0.166°, TT-TT: 6.43 ± 0.312°). This result was consistent with previous biomechanical studies [23, 34] and in lateral bending (CBT-CBT: 4.71 ± 0.718°, TT-TT: 7.19 ± 0.488°). This may be related to the differences in diameter and length between the TT and CBT screws. In terms of ROM of L4–L5 segment in CBT-TT and TT-CBT, there was a significantly lower ROM in CBT-TT compared to TT-TT, particularly in lateral bending (CBT-TT: 5.25 ± 0.510°, 27% lower and 4.69 ± 0.595°, 37% lower; TT-CBT: 5.40 ± 0.556°, 25% lower and 4.38 ± 0.795°, 41% lower in left and right lateral bending, respectively), while compared to the CBT-CBT group, the differences were not significant. This may be related to the increased holding strength of the vertebral body developed by different trajectories [35]. The ROM of posterior fixation has not been extensively discussed in previous studies [18–20]; nevertheless, the present study found that the ROM of CBT-TT and TT-CBT was significantly lower compared to both TT-TT and CBT-CBT, particularly in flexion (TT-TT: 1.860 ± 0.127°, CBT-CBT: 1.485 ± 0.055°, CBT-TT: 1.162 ± 0.042°, TT-CBT: 1.188 ± 0.144°) and extension (TT-TT: 2.380 ± 0.219°, CBT-CBT: 1.745 ± 0.060°, CBT-TT: 1.423 ± 0.063°, TT-CBT: 1.422 ± 0.078°). These differences were not significant in other conditions. This indicates that CBT-TT and TT-CBT have better resistance to activity in both flexion and extension. CBT-TT and TT-CBT displayed superior intervertebral disc stress dispersion ability in each condition, particularly in rotation. They effectively reduced the stress in the front of the intervertebral disc in flexion (TT-TT: 10.635 ± 0.567 MPa, CBT-CBT: 7.340 ± 0.515 MPa, CBT-TT: 5.995 ± 0.350 MPa, TT-CBT: 4.970 ± 0.370 MPa), while the stress at the back of intervertebral disc was effectively reduced in extension (TT-TT: 11.473 ± 0.243 MPa, CBT-CBT: 9.565 ± 0.241 MPa, CBT-TT: 6.690 ± 0.287 MPa, TT-CBT: 6.038 ± 0.310 MPa), which was clear in TT-CBT (Figure 6(b)). They effectively reduced the lateral stress of the intervertebral disc in lateral bending (TT-TT: 9.288 ± 0.395 MPa, CBT-CBT: 8.303 ± 0.370 MPa, CBT-TT: 6.080 ± 0.443 MPa, TT-CBT: 6.413 ± 0.513 MPa), and the intervertebral disc stress was concentrated in the central part in rotation, while at the same time, stress of the edge was dispersed (Figures 6(a) and 6(b)). Rastegar et al. [36] reported in a previous biomechanical study that cage subsidence has also been shown to be an important risk factor after lumbar interbody fusion. Lower cage stress might be obtained when decompression and fusion at the responsible stage is performed with the hybrid technique. In terms of posterior fixation stress, we found that the maximal von Mises stress of CBT-TT and TT-CBT was significantly lower than that of TT-TT, particularly in flexion and extension (CBT-TT: 62.825 ± 5.961 MPa, 38% lower and 61.240 ± 5.667 MPa, 40% lower; TT-CBT: 62.305 ±3.960 MPa, 36% lower and 66.350 ± 2.972 MPa, 40% lower in flexion and extension, respectively). Wang et al. [35] simulated the T12–L2 thoracolumbar 3D FE model with a fracture included in the L1 vertebra and demonstrated that, during cross-stage fixation, CBT-TT displayed a higher von Mises stress in lateral bending, but was lower in other conditions, compared to TT-TT. Interestingly, it showed a higher von Mises stress compared to CBT-CBT in each condition. In the present study, CBT-TT and TT-CBT displayed a lower von Mises stress in each condition compared to TT-TT and CBT-CBT, which may be related to the screw length, diameter, and moment arm length.

The stress distribution characteristics in the present study showed that the posterior fixation (e.g., screw and rod) has a clear restraint effect on the movement trend of the vertebral unit with the action of positive pressure and torque. Comparing the effect of different movement trends on the stress of the posterior fixation, it was found that the stress distribution of the screw inside the cancellous bone was superior to counterparts during flexion and extension, which was clear in TT-TT. The reason was that the direction of the movement trend was in the same plane as the axial direction of the screw and rod during flexion and extension. McLachlin et al. [37] found that early loose screws make use of the cortical bone as the fixation point, with their anterior end swinging in the cancellous bone, called the “teeter-totter” mechanism. In the present study, the cancellous thread area, anterior to the cortical thread, of TT-TT consistently displayed a higher von Mises stress distribution than its counterparts, which indicates that the use of a single application of TT or CBT screws was more prone to screw bone interface failure in accordance with the “teeter-totter” mechanism. By contrast, both the TT and CBT screws in the CBT-TT and TT-CBT groups displayed a lower von Mises stress distribution in this area (Figures 9(a) and 9(b)), which indicates a lower loosening rate of screws in the hybrid techniques. Interestingly, except for the area demonstrated above, the stress distribution for all fixations showed that the stress was concentrated near the screw hub (Figure 9), at the junction of the threaded and unthreaded regions, as reported by Chen et al. [38]. In the present study, we found that the hybrid techniques also probably reduce the von Mises stress in this area, particularly in flexion and extension. Apart from that, the stress of CBT screws was significantly concentrated posteriorly, and thus, the pars completeness was crucial to maintain the stability of the hybrid CBT-TT and TT-CBT techniques. Patients with a pars fracture may experience hybrid technique failure, such that this condition should be considered a relative contraindication for its use [37]. TT-CBT can be performed when there is pars fracture of the upper vertebral body. Therefore, this is why we proposed the hybrid TT-CBT technique as an ideal alternative for lumbar spondylolisthesis patients. In addition, as can be seen in Figure 9, CBT-TT and TT-CBT displayed a lower von Mises stress distribution of the rod in flexion and extension compared to their counterparts, which indicates that the hybrid techniques have a lower risk for rod breakage.

As with any FE analysis, certain limitations were inherent in the present study. First, there was a lack of ligaments and muscles, which play an important role in supporting the stability of the lumbar spine. Second, there was a lack of an adjacent segment which provides an indispensable role in evaluating the relationship between hybrid techniques and ASD. Third, linear elastic and homogeneous material properties for the vertebral body and the disc were lacking. Fourth, the limited number of specimens was insufficient to allow more convincing conclusions. Fifth, the rods in the hybrid techniques were not perpendicular to the horizontal line, but formed a certain included angle. From the stress nephograms of the hybrid techniques, it can be seen that the stress was reduced, but the force magnitude of the rod was not analyzed in considerable detail. Consequently, there is only one size of TT and CBT screws, thus the biomechanical effects of varies screw diameters and lengths in the hybrid techniques have not been considered extensively in the present literature. The present study did not standardize the sizes of the CBT and TT screws in the hybrid techniques.

## 5. Conclusion

Aim of this study is to provide posterior fixation with higher purchase and superior fixation strength. Among the different fixation techniques, CBT-TT and TT-CBT offered superior fixation strength, followed by CBT-CBT, while TT-TT was the least stable and resulted in the increased stress of the screws. Considering its superior segmental stability, the hybrid techniques might be effective in short segment fusion after limited spinal decompression or discectomy, particularly in elderly patients with osteoporosis. Hybrid techniques might be alternative in patients with pars fracture when CBT-CBT cannot be used. The results of this study reflected important factors to be considered in further biomechanical study, and more clinical studies with long-term follow-up are also necessary to validate the findings of the present study.

## Figures and Tables

**Figure 1:** Finite-element model of the lumber vertebra and diagrams illustrating the trajectory from the axial and sagittal views. (a) TT screws at the cranial and caudal levels (TT-TT); (b) CBT screws at the cranial and caudal levels (CBT-CBT); (c) CBT screws at the cranial level and TT screws at the caudal level (CBT-TT); (d) TT screws at the cranial level and CBT screws at the caudal level (TT-CBT); (e)–(h) are the axial and sagittal views of each respective technique of (a)–(d).

**Figure 2:** Displacement-load curves for the models and in vitro experiments. FE represents the results of the present study, while the remainder are the in vitro test results of Markolf [24], Virgin [25], and Brown et al. [26].

**Figure 3:** Mean values and minimum-maximum ranges of the ROM of L4–L5 segment for the models compared with the average and standard deviation of previous studies. FE refers to the current study.

**Figure 4:** Mean values and minimum-maximum ranges of the ROMs of the fixation segment in four implanted models. The maximum ROM was found for the TT-TT group, followed by the CBT-CBT, TT-CBT, and CBT-TT groups.

**Figure 5:** Mean values and minimum-maximum ranges of the ROMs of posterior fixations at the fixation segment in four implanted models. The maximum ROM was found for the TT-TT group, followed by the CBT-CBT, CBT-TT, and TT-CBT groups.

**Figure 6:** Stress nephograms over L4–L5 discs of the two different implanted models in flexion, extension, left lateral bending, right lateral bending, left rotation, and right rotation, respectively. The stress scales are the same in each condition. (a) Stress nephograms of CBT-TT. (b) stress nephograms of TT-CBT.

**Figure 7:** Mean values and minimum-maximum ranges of disc stresses at the fixation segment in four implanted models. The maximum disc stress was found for the TT-TT group, followed by the CBT-CBT, TT-CBT, and CBT-TT groups.

**Figure 8:** Mean values and minimum-maximum ranges of the peak von Mises stress in posterior fixations in four implanted models. The maximum stress was found for the TT-TT group in each condition, followed by the CBT-CBT, CBT-TT, and TT-CBT groups.

**Figure 9:** Stress nephograms of the posterior fixation of the two different implanted models in flexion, extension, left lateral bending, right lateral bending, left rotation, and right rotation, respectively. (a) Stress nephograms of CBT-TT. (b) stress nephograms of TT-CBT.

**Table 1:** Material properties of each component in the FE models.

Element	Element type	Modulus of elasticity (MPa)	Poisson ratio	Density (ton/mm^3^)
Vertebral cortical bone	C3D10M	12000	0.30	1.9*e* − 9
Vertebral cancellous bone	C3D10M	100	0.2	0.7*e* − 9
Annulus fibrosus and nucleus pulposus	C3D10M	3.2	0.45	0.9*e* − 9
Screw and rod	C3D10M	110000	0.3	4.5*e* − 9

## Data Availability

The biomechanical data used to support the findings of this study are included within the article.
